The article "Big Data and Learning Analytics Model for Promoting Physical Literacy in College Students in China" was retracted in 2023. Reasons: unreliable results or conclusions; concerns about the data; concerns about the peer review; concerns about the citations.

# Big Data and Learning Analytics Model for Promoting Physical Literacy in College Students in China

**DOI:** 10.1155/2021/8587351

**Published:** 2021-09-04

**Authors:** Yaping Zhao, Jie Cai, Lei Wang, Liang Zhao

**Affiliations:** ^1^Shandong Sport University, Jinan, China; ^2^Shandong University of Finance and Economics, Jinan, China; ^3^The School of Physical Education, Shandong University, Jinan, China

## Abstract

Physical literacy has gained much popularity in educational circles who are working on the improvement of curriculum and overall standard of education. It involves a holistic lifelong comprehensive learning approach that includes movements and physical activities. Overall, it has positive effects on physical, psychological, social, and cognitive health of individuals, so physical literacy exemplifies the dedication to raise a healthier, more active generation. Numerous factors interacting between humanities and social sciences affect the promotion of physical literacy, so such a study will be interdisciplinary which will consider across all social and individual factors. The current research proposes a system dynamic “SD” model to promote students' physical literacy by building a complete causal loop diagram of the model to illustrate the general system. Based on the casual loop diagram, the system is then presented as four subsystems. The model is simulated by allocating 14 different changes of indexes in the physical literacy promotion system to find better allocations for optimal effectiveness in promoting physical literacy. Simulations are carried out by using the Apache Spark architecture utilizing “Big Data” tools for effective, speedy, and reliable analysis and results. The study proposes that different physical literacy indexes in different grades require attention; the optimal promotion of physical literacy can be achieved by increasing the physical knowledge of lower-grade students and increasing the physical attitude of higher-grade students. The model can be used to make decisions about efficient physical literacy management and physical literacy promotion planning.

## 1. Introduction

Physical literacy is considered “the motivation, confidence, physical competence, understanding, and knowledge that individuals develop to maintain physical activity at an appropriate level throughout their life” ([1], p. 5). Physical literacy is a concept that has been developed over a long period of time. Although physical literacy may be thought of as a goal for a school-based physical education class, it is vital to remember that it is applicable throughout one's life. Six stages of physical literacy have been established in this regard, including infancy, childhood, adolescence, young, adulthood, and older adulthood.

The article "Big Data and Learning Analytics Model for Promoting Physical Literacy in College Students in China" was retracted in 2023. Reasons: unreliable results or conclusions; concerns about the data; concerns about the peer review; concerns about the citations.

The notion of physical literacy was introduced for the first time at the International Association of Physical Education and Sport for Girls and Women Congress in Melbourne, Australia in 1993 by Dr. Margaret Whitehead. The concept and definition of physical literacy were developed as a result of this research. Afterward, the implications of physical literacy as the objective of all structures were sketched out. The concept of physical literacy soon gained worldwide attention [2, 3], and many countries, like the United States (U.S.), the United Kingdom (U.K.), and Canada, promote physical literacy to encourage citizens to be active and healthy [4–6]. It is important to note that physical literacy has several advantages beyond physical health. Academic performance, cognitive skills, mental health, psychological well-being, social skills, and good lifestyle habits are all positively improved with physical literacy. As a result, it may be made mandatory for all the children to master fundamental movement and skills and develop physical literacy. Physical literacy is equally as important as reading and writing skills!

Research on physical literacy promotion has become increasingly popular [2], including a discussion on empowerment and its significance in promoting physical literacy [7]. Furthermore, Wang [8] researched the fusion method of Chinese traditional sports culture and physical literacy. However, these studies only addressed theoretical analysis, i.e., they lacked effective methods and supporting data.

On the other hand, some studies presented promotional strategies for different groups, for example, Zhang and Dong [9] researched the connotation and promotion path of university students' physical literacy. Moreover, JungHwanCho [10] discussed the importance of physical literacy promotion and suggested potential implementation strategies specific to the life stages of special population groups in the Korean context. Furthermore, Savelsbergh and Wormhoudt [11] presented an athletic skills model as a suitable framework to structure (developmental) movement programs to enhance physical literacy. Although they used some effective methods to promote physical literacy, the means to allocate strategies to promote physical literacy most effectively have rarely been discussed.

Forrester [12] established a system dynamics (SD) model to study the behaviors of feedback loops, which contained stocks (levels) and flows. SD provides an effective way for modeling, simulating, and researching complex systems and had been applied in many fields, including management, economics, and transportation. For instance, Zhou et al. [13] established an SD model to solve a third-party logistics inventory problem, and Duan et al. [14] proposed an SD model to verify a human resource management strategy. Furthermore, Olaya et al. [15] built an SD model using De Soto's theory of an informal economy, while BenDor [16] analyzed the dynamics of U.S. automobile gasoline consumption since 1975 with an SD model. Furthermore, Ercan et al. [17] used an SD approach to model and simulate the most realistic and practical carbon dioxide mitigation scenarios for U.S. cities by adopting future public transportation policies.

The article "Big Data and Learning Analytics Model for Promoting Physical Literacy in College Students in China" was retracted in 2023. Reasons: unreliable results or conclusions; concerns about the data; concerns about the peer review; concerns about the citations.

To the best of our knowledge, little research has employed an SD model on physical literacy promotion in China. Although some promotional strategies were studied and implemented, evaluating and maximizing the effectiveness of those strategies is a complex task that needs proper attention. SD is an effective way to address this problem [18]. Therefore, this study is focused towards the development of an SD model for physical literacy promotion to determine a better allocation for achieving promotion effectiveness. The current study relies on the usage of big data analysis tools which are proved to be very successful in predictive analysis and in user behavior study systems. These systems can consume data sets of any size and complexity and can effectively capture discriminating information, formulate better feature sets, present better analysis, and yield effective visualization and querying. The current study utilizes the advantages of big data by using Apache Spark Hadoop services, which is open-source software for reliable, scalable, distributed computing. This will not only provide effective simulation results but also ensures better reliability, speed, and precision due to its distributed working mechanism. In the subsequent section, we will discuss four cases and their specific simulations to illustrate the results.

## 2. The SD Model

### 2.1. Causal Relationship of Students' Physical Literacy Promotion

The whole system of physical literacy consists many subsystems but to simplify the analysis; we posited that there are four subsystems: physical knowledge, physical skill, physical attitude, and physical competence. Based on the introduction of problems and impacts in the physical literacy promotion system [19] discussed before, the entire causal loop diagram for the system is shown in Figure 1.

To explain the proposed model, we used two loops.

“Physical literacy⟶−self-knowledge satisfaction⟶−physical knowledge⟶+physical literacy.”

“Physical literacy⟶+fitness burnout⟶−physical skill⟶−physical literacy.”

The first is a positive feedback loop where by increasing physical literacy, the degree of self-knowledge satisfaction is reduced. The lower degree of self-knowledge satisfaction will lead to increased physical knowledge due to more active learning actions [20], which have a positive impact on the physical literacy itself. The second loop is a negative feedback loop, that is, an increase in the first parameter will increase the feeling of fitness burnout, leading to a lower degree of physical skill, which will ultimately reduce the physical literacy.

The article "Big Data and Learning Analytics Model for Promoting Physical Literacy in College Students in China" was retracted in 2023. Reasons: unreliable results or conclusions; concerns about the data; concerns about the peer review; concerns about the citations.

### 2.2. Flow Diagram of the Physical Literacy Promotion Subsystem

To sketch the flow diagram of the physical literacy promotion subsystem, following assumptions are made: (1) It is assumed that the four subsystems are interdependent and independent of each other in order to illustrate the results more clearly. Being a common parameter in each subsystem, the physical literacy is influenced by all the subsystems but to simplify the mathematical modeling of subsystems, it is anticipated that physical literacy is determined only by this particular subsystem and not influenced by other subsystems. (2) To reflect the reality of college students, we assumed a total duration of three years from being a freshman to being a senior. (3) The implementation of physical literacy promotion measures for college students has been increasing in schools and society; thus, it is assumed that the resources and environments associated with students' physical literacy changed over time. (4) To simplify the model and match the facts, the negative variation caused by disease and accidental injury was ignored [21], and system collapse caused by major changes and other abnormal situations was not considered.

Based on the analysis of the causal relationship of students' physical literacy promotion, four subsystems are established as explained in the following subsections. Six experts in physical activity and literacy, two doctoral tutors, and four PhDs evaluated all the coefficients.

#### 2.2.1. Physical Knowledge

Physical knowledge is the state variable, where physical knowledge reduction and increase are the variable's rate determined by physical knowledge increase minus physical knowledge reduction. Physical knowledge reduction comprises self-knowledge satisfaction, and the degree of physical literacy affects self-knowledge satisfaction [22]. The higher the physical literacy, the higher the thirst for knowledge and decreasing self-knowledge satisfaction. Knowledge source is a time-dependent variable, as with the development of civilization and information technology, more knowledge can be obtained. To express this, following equations are formulated:

(1) $$\begin{array}{c} \text{physical knowledge}=\text{physical knowledge increase}-\text{physical knowledge reduction},\\ \text{physical knowledge reduction}=0.8*\text{self}-\text{knowledge satisfaction},\text{physical knowledge reduction}=0.8*\text{self}-\text{knowledge satisfaction},\\ \text{self}-\text{knowledge satisfaction}=2-0.1*\text{physical literacy},\\ \text{physical knowledge increase}=\text{learning ability}\left(\text{knowledge source}\right). \end{array}$$

The article "Big Data and Learning Analytics Model for Promoting Physical Literacy in College Students in China" was retracted in 2023. Reasons: unreliable results or conclusions; concerns about the data; concerns about the peer review; concerns about the citations.

#### 2.2.2. Physical Skill

Physical skill is the state variable, where physical skill enhancement and skill decrease are the vaiable's rate determined by physical skill enhancement minus physical skill decrease. Physical skill decrease comprises fitness burnout, and the degree of physical literacy affects fitness burnout [23]. According to Zhao [19], higher physical literacy leads to satisfaction with one's current skill level. The fitness environment is a time-dependent variable because the increase in national support has constantly improved the fitness environment. To express this, following equations are formulated:

(2) $$\begin{array}{c} \text{physical skill}=\text{physical skill enhancement}-\text{physical skill decrease},\\ \text{physical skill decrease}=0.7*\text{fitness burnout},\\ \text{fitness burnout}=0.2*\text{physical literacy},\\ \text{physical skill enhancement}=\text{professional guidance}\left(\text{fitness environment}\right). \end{array}$$

#### 2.2.3. Physical Attitude

Physical attitude is the state variable, where physical attitude diminishment and enhancement are the variable's rate. Physical attitude is calculated as physical attitude enhancement minus physical attitude diminishment. Physical attitude diminishment comprises other temptations since the degree of physical literacy affects other temptations. Owing to increased knowledge and skill promoting attitude enhancement, physical attitude enhancement is influenced by physical knowledge increase and physical skill enhancement [24, 25]. Learning attitude is a time-dependent variable, varying over time. Therefore, the following equations are formulated:

(3) $$\begin{array}{c} \text{physical attitude}=\text{physical attitude enhancement}-\text{physical attitude diminishment},\\ \text{physical attitude diminishment}=0.5*\text{other temptations},\\ \text{other temptations}=2+0.1*\text{physical literacy},\\ \text{physical attitude enhancement}=\text{excitation}\left(\text{learning attitude}\right)+0.27*\text{physical knowledge increase}+0.22*\text{physical skill enchancement}. \end{array}$$

#### 2.2.4. Physical Competence Subsystem

Physical competence is the state variable, where physical competence improvement and debasement are the variable's rate. The physical competence debasement is affected by the lack of motivation, and the degree of physical literacy affects the lack of motivation [26]. Since the increase in knowledge and attitude promote competence [27], physical competence improvement is influenced by physical knowledge increase and physical attitude enhancement. Fitness atmosphere is a time-dependent variable since the fitness atmosphere improves as the public pays more attention to fitness. To express this, we used the following equations:

(4) $$\begin{array}{c} \text{physical competence}=\text{physical competence improvement}-\text{physical competence debasement},\\ \text{physical competence debasement}=0.8*\text{lack of motivation},\\ \text{lack of motivation}=1+0.1*\text{physical literacy},\\ \text{physical competence improvement}=1.25*\text{self}-\text{control}\left(\text{fitness atmosphere}\right)+0.38*\text{physical knowledge increase}+0.29*\text{physical attitude enhancement}. \end{array}$$

The article "Big Data and Learning Analytics Model for Promoting Physical Literacy in College Students in China" was retracted in 2023. Reasons: unreliable results or conclusions; concerns about the data; concerns about the peer review; concerns about the citations.

### 2.3. General System Flow Diagram of Students' Physical Literacy Promotion

Based on the aforementioned analysis, the general system flow diagram of physical literacy promotion of college students in China is presented in Figure 2.

The four subsystems are combined with the “physical literacy” variable where the Cobb–Douglas production function is utilized to evaluate physical literacy. The Cobb–Douglas production function predominantly deals with the relationship between changes in the quantities of various elements and with the output produced within a certain period using the same technical level [28]. It is a mathematical model used to predict the production of industrial systems in countries/regions and is one of the most widely used production function in economics [29].

The current study on physical literacy explored the relationship between the variables contained in the four major subsystems while assuming that the external variables remain unchanged. The assumption about the relationship between the dependent and independent variables is consistent with the classic analysis model of the Cobb–Douglas production function applicable to the analysis of the contribution rate of changes in factors to output. Consequently, this study abstracts the degree of physical literacy as the output of the four major subsystems and describes it with the classic Cobb–Douglas production function. All coefficients were evaluated by research group experts and were consistent with the subsystem equations.

(5) $$\begin{array}{c} \text{physical literacy }=\text{ physical knowledge }\left(\text{0.}17\right)*\text{physical skill}\left(\text{0.}28\right)*\text{physical attitude}\left(\text{0.}25\right)*\text{physical competence}\left(\text{0.}3\right). \end{array}$$

The article "Big Data and Learning Analytics Model for Promoting Physical Literacy in College Students in China" was retracted in 2023. Reasons: unreliable results or conclusions; concerns about the data; concerns about the peer review; concerns about the citations.

## 3. Materials and Methods

An Institutional Review Board approval was not required for this study as the data used are obtained from existing literature and accordingly, the SD method was used to simulate the data. This study does not involve a questionnaire survey or human experiments. In the implementation, the simulation was initialized as INITIAL − TIME = 0, FINAL − TIME = 36, TIME − STEP = 1, where the time unit is months.

### 3.1. Benchmark Dataset

The current study presents a case study of physical literacy promotion among college students in China where the utilized data are captured by Zhao [19] and a physical education school in Shandong University, China. The SD model is based on the actual data from students in each college grade. The data of freshmen is the initial data in the SD model, while the data of sophomores are the data of the 12th month in the SD model. Similarly, the data of junior students is the data of the 24th month in the SD model, and the data of senior students are the final data in the SD model [30]. The specific initial variables are presented in Table 1. Based on the data, further degree of physical literacy of each grade is calculated as presented in Table 2.

### 3.2. Methods

The proposed model is studied by examining it across different tests elaborated in the following subsections:

#### 3.2.1. Appearance Test

An appearance test is used to determine whether the model structure is consistent with the actual situation [31]. In the SD model of physical literacy, the research group experts evaluated all the coefficients and found the model consistent with the actual situation.

#### 3.2.2. Operation Test

An operation test is performed by observing whether there is any ill-result output in operating the model [32]. Different simulation steps are selected in this test where the chosen step sizes are set to 0.25, 0.5, and 1. The whole operation process is found to be stable, yielding no ill results.

#### 3.2.3. Historical Test

A historical test identifies the difference between simulation results and actual data to ensure that the model is consistent with reality [33]. Owing to a historical test of the simulation data of physical knowledge, physical skill, physical attitude, physical competence, and physical literacy, the error between the simulation result and the actual result is observed to be less than 5%.

#### 3.2.4. Sensitivity Test

A sensitivity test is performed to compare the simulation results by changing the structure, equation, or parameters of the established model and observing the impact in the amount of change in the system [34]. A sensitivity test is generally divided into parameter sensitivity and structure of sensitivity. Professional guidance is selected as the variable to conduct a sensitivity test. In current scenario, 3% reduction or 3% increase in the parameter of professional guidance indicates that there are no significant changes. Similarly, in the structure sensitivity test, the relationship of the SD model remains clear, and the structure proved to be effective through literature support and theoretical analysis.

The article "Big Data and Learning Analytics Model for Promoting Physical Literacy in College Students in China" was retracted in 2023. Reasons: unreliable results or conclusions; concerns about the data; concerns about the peer review; concerns about the citations.

### 3.3. Simulations

For simulation purpose, four indexes are selected, including physical knowledge increase, physical skill enhancement, physical attitude enhancement, and physical competence improvement, which served as the control parameters for simulation control. The four indexes can change with time and be influenced by government and society. For better projection and evaluation, three models are designed by changing one index, two indexes, and three indexes, respectively, as depicted in Table 3. The corresponding simulation results are presented in Figures 3–5. In the end, important node data are presented in Table 4 for better observation.

## 4. Design of the Proposed Model

This section discusses the design of the suggested model along with all its subsidiary components.

### 4.1. Apache Spark Architecture

Apache Spark is an open-source system, which provides unified analysis services for large-scale data processing. It provides an interface to program full cluster with implicit data parallelism and fault tolerance. The overall architecture of Spark in a distributed environment is shown in Figure 6, which mainly includes two modules: Driver and Worker. The Driver creates SparkContext by running the main method in the application, creates the Resilient Distributed Dataset (RDD), and performs the corresponding transformation actions on the RDD. SparkContext serves as a bridge between the data processing logic and the Spark cluster and is responsible for communicating with ClusterManager. ClusterManager makes unified scheduling of the cluster's resources and allocates required cluster computing resources for the task as well as launches Executor to improve the efficiency of task scheduling as much as possible. The work of computing Tasks in the cluster is taken care of by the WorkNode. When a computing task is executed on a cluster, the WorkNode starts an Executor for the Task. Then, the Executor starts a thread pool that manages the Task, which acts as the unit of computation on the Executor. The Driver will receive information from the Executor about the health of the Task, and finally, the Executor will stop when all tasks have been executed. In addition, after years of accumulation, Spark has a series of components that constitute its ecosystem [35]. The Spark core composition is shown in Figure 7.

The article "Big Data and Learning Analytics Model for Promoting Physical Literacy in College Students in China" was retracted in 2023. Reasons: unreliable results or conclusions; concerns about the data; concerns about the peer review; concerns about the citations.

The SparkCore is the cornerstone and core of the entire Spark ecosystem, which mainly includes the creation of SparkContext, storage system, basic model architecture, task running process, and calculation engine. Spark SQL completes the processing function of structured data, and Spark Streaming can complete the function of real-time calculation, providing users with functions, such as real-time data collection, real-time data calculation, and real-time data query. GraphX is a distributed graph computing processing tool provided by the Spark platform, which can be deployed in a distributed cluster. The framework has a rich graph computing mining API. Finally, MLib is a Spark machine learning component that makes machine learning easier to implement, and it also facilitates the processing of larger-scale data.

## 5. Experiments and Results

The following sections present the simulation environment and discusses the outcomes with supportive reasoning.

### 5.1. Experimental Environment

The experimental environment of Apache Spark as configured for the current study is presented in Table 5.

For the experimentation purposes, a Spark cluster is built, utilizing 5 physical processing nodes with default settings. The essential hardware and software requirements employed throughout the tests are explained in Table 5. All processing nodes are operated using the Ubuntu 18 LTS operating system, Spark 2.3.4, and Hadoop 2.7.3. The remaining three nodes were set up as the working nodes for the master node.

The results revealed that in the first model, when only one index was changed, at month 12 (i.e., sophomore), the change in the physical knowledge index played the largest role in improving physical literacy, while the changes in the physical attitude and physical competence indexes had similar effects. On the other hand, the change in the physical skill index was the least effective. At month 24 (i.e., junior), the change in the physical knowledge index played the largest role in improving physical literacy, followed by the changes in the physical attitude and physical competence indexes. The change in the physical skill index still played a minimal role. At month 36 (i.e., senior), the change in the physical attitude index played the largest role in improving physical literacy, followed by the changes in the physical knowledge and physical skill indexes. Contrary to earlier time points, the change in the physical competence index played a minimal role at this stage.

The article "Big Data and Learning Analytics Model for Promoting Physical Literacy in College Students in China" was retracted in 2023. Reasons: unreliable results or conclusions; concerns about the data; concerns about the peer review; concerns about the citations.

In the second model, where two indexes are changed at a time, for instance, at month 12 and month 24, the changes in both the physical knowledge and physical attitude indexes played the largest roles in improving physical literacy, while the changes in both the physical skill and physical competence indexes impacted physical literacy the least. At month 36 (i.e., senior), the changes in both physical skill and physical attitude indexes improved physical literacy the most, whereas the changes in the physical knowledge and physical competence indexes had the least effect on improving physical literacy.

In the third model, as depicted in Table 3, where three indexes are changed simultaneously, the changes played important role in improving physical literacy significantly.

In sum, to obtain a more effective promotion of physical literacy with a single index, the physical knowledge of the lower-grade students needs to be significantly increased, while for higher-grade students, an increase in physical attitude made the greatest contribution to the promotion of physical literacy. To obtain a more effective promotion of physical literacy with two indexes, physical knowledge and physical attitude become the candidate parameters to be increased for lower-grade students, while for higher-grade students, an increase in both the physical skill and physical attitude indexes made the greatest contribution to the promotion of physical literacy. In the end, an increase in all the indexes results in a more overall effective promotion of physical literacy.

## 6. Discussion

The current study presented an SD model for promoting physical literacy among college students in China to determine a better allocation for obtaining the most effective promotional strategy. The results showed that different physical literacy indexes need attention at different grades, i.e., for lower-grade students, the increase in the physical knowledge index played the most important role in the promotion of physical literacy, whereas for higher-grade students, the increase in physical attitude index had the best effect in promoting physical literacy.

The findings of the current research significantly contributed to the extant literature on this topic. First, the objective of previous studies mainly introduced the empowerment and significance of promoting physical literacy and employed distinct strategies for different groups. These studies would be more meaningful if targeted towards solving specific problems instead of talking about physical literacy promotion in general. Therefore, in this study, our objective was to solve a specific problem, i.e., finding a better allocation to obtain the best method in order to promote physical literacy.

The article "Big Data and Learning Analytics Model for Promoting Physical Literacy in College Students in China" was retracted in 2023. Reasons: unreliable results or conclusions; concerns about the data; concerns about the peer review; concerns about the citations.

Secondly, the current study suggests the suitability of using the SD method to establish a general model. SD is a method of modeling that ignores the details of a system and produces a general representation of a complex system. It has been widely used in strategic and policymaking modeling and simulation in fields, such as management [14], economics [15, 16], and transportation [17]. Thus, compared with other related research results, the results presented in current study have more theoretical value and practical significance.

Lastly, most of the other researches mainly conducted qualitative and theoretical analyses and failed to use effective methods or data to support their claims. To overcome this limitation in current work, an SD model is employed where a real case is presented, making the study and results more convincing.

Despite these strengths, this paper also has some limitations. The simulation results in this paper are based on the present scenarios. For the sake of analysis, we did not consider all possible scenarios, such as sudden illness or natural disasters. For the comparison, we only chose 14 cases. In the future, more parameters may be considered, which can affect physical literacy as well as subsequent cases to verify the efficacy of the proposed model and to determine the best cases and strategies in order to improve physical literacy as well as to make the model more promising.

## 7. Conclusion

This paper presented an SD model for the promotion of physical literacy among college students in China. The physical literacy promotion is regarded as a whole system, which is divided it into four subsystems: physical knowledge, skill, attitude, and competence, where the objective was to find a better allocation for ideal promotion effectiveness of physical literacy. The model is tested on 14 different allocations of changes in the indexes of the physical literacy promotion system. The results suggest that paying attention to different physical literacy indexes at different college levels can significantly promote physical education where the physical literacy can be best achieved by increasing the physical knowledge of lower-grade students and the physical attitude of higher-grade students. Due to nonavailability of data, the study is limited to college students only, but as a future prospect, it is recommended to extend this study for school going youngsters, which will further extend the benefits of this research.

## Figures and Tables

**Figure 1:** A complete causal loop diagram of the system.

**Figure 2:** Flow diagram of the general system.

**Figure 3:** Simulation results of model 1.

The article "Big Data and Learning Analytics Model for Promoting Physical Literacy in College Students in China" was retracted in 2023. Reasons: unreliable results or conclusions; concerns about the data; concerns about the peer review; concerns about the citations.

**Figure 4:** Simulation results of model 2.

**Figure 5:** Simulation results of model 1.

**Figure 6:** Spark's overall architecture [35].

**Figure 7:** The core composition of Spark [35].

**Table 1:** The main parameters in the model.

Variable	Initial value			
	Freshman	Sophomore	Junior	Senior
Physical knowledge	4.03	4.11	4.05	3.78
Physical skill	4.01	4.20	4.07	3.78
Physical attitude	3.28	3.55	3.46	3.14
Physical competence	3.42	3.61	3.40	2.94

**Table 2:** The degree of physical literacy of each grade.

Grade	Physical literacy
Freshman	3.63
Sophomore	3.83
Junior	3.70
Senior	3.35

**Table 3:** The four regulatory schemes in models 1, 2, and 3.

Regulatory schemes	Physical literacy	Physical knowledge increase	Physical skill enhancement	Physical attitude enhancement	Physical competence improvement
Model 1	Case 1	3% growth	No change	No change	No change
	Case 2	No change	3% growth	No change	No change
	Case 3	No change	No change	3% growth	No change
	Case 4	No change	No change	No change	3% growth
Model 2	Case 5	3% growth	3% growth	No change	No change
	Case 6	3% growth	No change	3% growth	No change
	Case 7	3% growth	No change	No change	3% growth
	Case 8	No change	3% growth	3% growth	No change
	Case 9	No change	3% growth	No change	3% growth
	Case 10	No change	No change	3% growth	3% growth
Model 3	Case 11	3% growth	3% growth	3% growth	No change
	Case 12	3% growth	3% growth	No change	3% growth
	Case 13	3% growth	No change	3% growth	3% growth
	Case 14	No change	3% growth	3% growth	3% growth

**Table 4:** The degree of physical literacy of each grade.

Grade	Month 0	Month 12	Month 24	Month 36
Actual	3.63	4.02	3.70	3.35
Case 1	3.65	4.14	4.11	3.65
Case 2	3.65	4.07	4.04	3.64
Case 3	3.65	4.11	4.09	3.66
Case 4	3.65	4.11	4.07	3.62
Case 5	3.65	4.16	4.19	3.77
Case 6	3.65	4.21	4.22	3.74
Case 7	3.65	4.20	4.20	3.71
Case 8	3.65	4.14	4.17	3.78
Case 9	3.65	4.13	4.15	3.74
Case 10	3.65	4.18	4.19	3.73
Case 11	3.65	4.26	4.31	3.85
Case 12	3.65	4.26	4.29	3.82
Case 13	3.65	4.23	4.28	3.84
Case 14	3.65	4.36	4.41	3.87

**Table 5:** Apache Spark configuration details of the cluster.

Specification	Processor	3.20 GHz *×* 10
	Connectivity	100 Mbps Ethernet LAN
	Hard disk	1 TB
	Memory	250 GB
	CPU	Intel Core Tm

Software	Operating system	Ubuntu 18 LTS
	Hadoop	2.7.3
	OS type	64 bit
	Spark	2.3.4
	Java Development Kit	16

## Data Availability

The data used to support the findings of this study are included within the article.
